# Moth-Flame Optimization for Early Prediction of Heart Diseases

**DOI:** 10.1155/2022/9178302

**Published:** 2022-09-12

**Authors:** S. Haseena, S. Kavi Priya, S. Saroja, R. Madavan, M. Muhibbullah, Umashankar Subramaniam

**Affiliations:** ^1^Department of Information Technology, Mepco Schlenk Engineering College, Sivakasi, India; ^2^Department of Computer Science and Engineering, Mepco Schlenk Engineering College, Sivakasi, India; ^3^Department of Electrical and Electronics Engineering, P.S.R Engineering College, Sivakasi, India; ^4^Department of Electrical and Electronic Engineering, Bangladesh University, Dhaka 1207, Bangladesh; ^5^Renewable Energy Laboratory, College of Engineering, Prince Sultan University, Riyadh, Saudi Arabia

## Abstract

Heart disease is among the leading causes of mortality globally. Predicting cardiovascular disease is a major difficulty in clinical data analysis. AI has been demonstrated to be powerful in deciding and anticipating an enormous measure of information created by the health domain. We provide a unique method for finding essential traits employing machine learning approaches in this paper, which enhances the effectiveness of identifying heart diseases. Decision tree (DT), support vector machine (SVM), artificial neural network (ANN), and K-nearest neighbor (KNN) are the classification techniques used to create the proposed system. Ensemble stacking integrates the four classification models to create a single best-fit predictive model using logistic regression. Many explorations have been directed at the identification of cardiac infection; however, the exactness of the outcomes is poor. Accordingly, to further enhance the efficiency, Moth-Flame Optimization (MFO) algorithm is proposed. The feature selection strategies are used to improve the classification accuracy while shortening the execution time of the classification system. Medical data are used to assess the probability of heart disease based on BP, age, gender, chest ache, cholesterol, blood sugar, and other variables. Results revealed that the proposed system excelled other existing models, obtaining 99% accuracy in the Cleveland dataset.

## 1. Introduction

Heart disease refers to a group of illnesses that affect people's hearts and veins. The symptoms of cardiac disease differ from person to person [1]. Cardiac disease alludes to a bunch of issues characterized by side effects, for example, hypertension, stroke, respiratory failure, and arrhythmia. The trouble for medical services suppliers is to give top notch care at a reasonable cost. Inadequate outcomes may result from an inaccurate clinical diagnosis and poor therapy. Detecting and diagnosing cardiovascular illness is a never-ending task that can be accomplished by a skilled practitioner with significant experience and understanding [2]. Decision support systems (DSSs) may be used by healthcare organizations to cut costs [3]. Patient records, various disease diagnoses, resource management, and other aspects of healthcare are common.

There has been a lot of work put into establishing remote monitoring gadgets and processes for diagnosing patients. Device exhaustion, then again, has been viewed as a hindrance to adherence [4]. Commercially accessible technologies have been exhibited to conquer this boundary by lessening the necessity for human contact [5], and the precision of action trackers has been shown to be adequate for health workers [6]. Clinical records are continually being produced, processed, and evaluated as a result of the advent of information technology systems. Clinical reports contain data that could be utilized to develop new healthcare services around the world, addressing issues such as social and economic status. Clinical reports, for example, contain a variety of numerical data, medical descriptions, images, etc. All of which can be used to create content-based services to help patients and doctors.

Rapid cardiovascular disease diagnosis of high-risk patients and faster detection using a prediction system has been widely proposed to reduce mortality rates and improve selection for future diagnosis and interventions [7]. A decision support system (DSS) framework may be utilized to assist clinicians in assessing the chance of cardiovascular problems and providing suitable medicines to further prevent the occurrence. Moreover, several studies have indicated that adopting a DSS can enhance preventive services, treatment planning, and better decision-making [8]. An expert DSS based on machine learning (ML) model and metaheuristics approach is used to efficiently identify heart disease.

The ML prescient models need legitimate information for preparing and testing. ML is now being utilized in hospitals to aid in the organization of administrative procedures, the planning and management of infectious diseases, and the customization of medical treatments [9]. Besides, the machine is presently utilized in an assortment of heart-related disciplines, as well as the improvement of new medical operations, the control of patient information and records, and the therapy of persistent illnesses [10, 11].

Supervised method [12] is an ML approach that predicts future data by mapping data flow based on labeled training information. The goal of this approach is aimed at creating a model and then improving the machine's performance as it is exposed to new data. Unsupervised learning technique is an ML method in which the system is given an unlabeled dataset and is required to uncover relationships within the data. Unsupervised learning is aimed at grouping data together and detecting existing patterns. Reinforcement learning algorithm uses trial and error to uncover the pattern or relationship within the data. An agent who makes decisions, the environment in which the agent interacts, and the actions that the agent must complete are the three key components involved. This algorithm's purpose is to discover the optimum policy based on experience to make reliable decisions.

Data mining and machine learning (ML) approaches minimize computer costs and time. One use of ML is the detection of medical disorders and therapies to enhance a patient's quality of life. Heart disease is commonly thought to be a condition that only affects the elderly; nevertheless, it is growing more common in people of all ages.

Information preprocessing is expected for information standardization to further develop ML models' expectation capacities. Preprocessing techniques such as noisy data removal and normalization are carried out. Model performance is also improved by feature extraction and selection strategies. Feature selection is performed using Moth-Flame Optimization technique and feature extraction using principal component analysis. Furthermore, classification is performed using four models, namely, DT, SVM, ANN, and KNN. Ensemble stacking is performed to combine the results from four classification models using logistic regression. The proposed system's result is evaluated using several metrics such as accuracy, precision, recall, and *F*-measure.

The main contributions of this research include the following:

- An automated system is designed to classify the dataset using Cleveland dataset
- Feature selection is performed using Moth-Flame Optimization algorithm that helps in removing unwanted features present in the dataset
- Feature extraction is carried out using principal component analysis (PCA) that helps in reducing the dimensionality of the dataset further
- Classification is performed using four different models, and the best results are obtained using the ensemble stacking method
- The system outperforms the existing state-of-art systems concerning accuracy, precision, recall, and *F*-measure

The following shows the breakdown of this intended work.  Section 2 goes into detail on the work related to the planned task.  Section 3 goes into detail about the proposed framework. The fourth section digs into the specifics of experimental outcomes and performance evaluation.  Section 5 discusses the conclusion as well as future efforts.

## 2. Literature Works

Researchers have proposed several ML-based diagnostic methodologies for HD. ML algorithms [13, 14] have been extensively utilized in a variety of research such as disease recognition and identification [15]. Gudadhe et al. [16] used multilayer perceptron and SVM to create a detection approach for heart disease (HD) categorization, which achieved an efficiency of 81%. Detrano et al. [17] used ML classification techniques to construct the HD classification system, which had 77 percent accuracy.

Al-Makhadmeh and Tolba [18] introduced a deep belief neural network model-based IoT-based heart disease identification system. The collected data was examined for missing values. The writers looked at how the data was distributed. The authors also employed the studentized approach to use normalized data. Deep belief networks and a high-order Boltzmann machine were used to extract features from noiseless data to be used by the model. The researchers achieved a prediction accuracy of 99.03, which can aid in the reduction of heart disease mortality. Ahmed [19] proposed an HD identification algorithm employing IoT architecture with SVM. To forecast heart disease, the patient data was analyzed using an SVM. The researchers claim that their method predicted cardiac disease with 97.53 percent accuracy. Using an IoT device, they acquired heart data and identified HD. This method detected HD in a short period of time, but the accuracy suffered when a large amount of data was used [20].

Guidi et al. [21] helped to create a DSS for heart failure analysis (HF). They investigated the effectiveness of neural networks (NN), SVM, CART-based fuzzy rules, and random forests, among other ML classifiers (RF). The CART model with random forests produced the best results, with an accuracy of 87.6 percent. Parthiban and Srivatsa [22] explored an SVM approach for detecting HD in diabetic patients with an efficiency of 95%.

Melillo et al. [23] led to the formation of an automated classification model that differentiates between those at low and high risk. The sensitivity and specificity of the classification and regression tree (CART) were calculated to be 93.3 percent and 63.5 percent, respectively. To reduce the number of features, Sewak et al. [24] employed a binary classifier that correctly identified heart disease with a 100% improvement in accuracy. Various techniques are available for feature selection [25, 26]. PCA [27, 28] has been employed as a feature retrieval strategy for categorization in healthcare services in recent research.

Classification is performed using Cleveland dataset [29] to identify if a patient had heart disease or not. The ML algorithms combined with feature extraction have three major goals: (i) to discover the unique features, (ii) evaluate the efficiency of PCA, and (iii) investigate the model that produces better results.

## 3. Proposed Methodology

This section describes the proposed system and its components in detail.  Figure 1 depicts the proposed system's schematic diagram.

### 3.1. Materials

In this research, the Cleveland dataset is used. There were 303 occurrences and 75 features when this dataset was designed. We preprocessed the dataset in this research, and six samples were excluded due to missing values in this dataset.

### 3.2. Data Preprocessing

Data preparation is a crucial stage in ML that enhances the quality of the data and makes it easier to extract useful knowledge from big data. Data preprocessing is a method of organizing and managing unprocessed data to prepare it for the development and training of ML models. Data cleaning is the process of eliminating erroneous, missing, and inconsistent data from databases as well as restoring missing data. After 6 samples with missing values are discarded, the remaining samples are processed. The absence and the presence of HD are portrayed by a solitary result marked with two classes. After missing values are eliminated, the data should be normalized well within the range from 0 to 1 to make evaluating heart disease trends easier. The studentized residual methodology is a standard deviation computation-based normalizing method [30]. To standardize the data for HD prediction, several data distributions and regression analysis are employed.

### 3.3. Dimensionality Reduction

The process of lowering the variables analyzed is known as dimensionality reduction [31]. It is employed to retrieve hidden characteristics within the unprocessed without sacrificing the integrity. This work incorporates 2 methods: the Moth-Flame Optimization (MFO) [32] for feature selection and the principal component analysis (PCA) for feature extraction [33].

#### 3.3.1. Feature Selection by Moth-Flame Optimization (MFO) Algorithm

MFO is an optimization approach focused on moths' use of transverse orientation to travel at night. Moths may fly greater ranges in a linear fashion by keeping a constant alignment towards the Moon. When moths come into touch with ambient light, they strive to maintain the same angle towards the light source, but the close closeness causes them to become entangled in a spiral route.

The MFO method distributes moths to various alternatives in the optimization problem's solution space, within each fitness function. Every moth carries a flame containing the optimal solution the moth has discovered. The moths fly in a circular route around their flames, changing their locations in each iteration as they explore the solution space. In MFO, moth positions are randomly set inside the solution space. The moths' fitness values are calculated. Each moth's best individual location is identified by the flame. The flame identifies the ideal location for every moth. The moths' locations are improved using a spiral movement algorithm nearing their best individual positions highlighted by a flame in the following iteration, and the flames' locations are replaced with new optimum and most consistent locations. Until the termination requirements are reached, the MFO algorithm keeps updating and generating new positions for the moths and flames.

The following is the computing procedure for MFO:

**Step 1 (creating the preliminary population).**

Each moth is considered to occupy a *P*-dimensional solution space. The collection of moths might be written as

(1) $$\begin{array}{c} N=\left[\begin{array}{ccc} N_{1,1}\; & \cdots & N_{1,p}\;\\ N_{2,1} & \cdots & N_{2,p}\\ \vdots & \ddots & \vdots \\ \;N_{m,1}\; & \cdots & N_{m,p} \end{array}\right], \end{array}$$

where *m* denotes the moth and *p* denotes the dimensions. The fitness function is given by

(2) $$\begin{array}{c} F=\left[\begin{array}{c} f_{1}\\ f_{2}\\ \vdots \\ f_{m} \end{array}\right]. \end{array}$$

Two components of the MFO include flames and their respective fitness functions as shown below:

(3) $$\begin{array}{c} FM=\left[\begin{array}{ccc} {FM}_{1,1}\; & \cdots & {FM}_{1,p}\\ {FM}_{2,1} & \cdots & {FM}_{2,p}\\ \vdots & \ddots & \vdots \\ {FM}_{m,1}\; & \cdots & {FM}_{m,p} \end{array}\right],\\ \text{OF}=\left[\begin{array}{c} {\text{of}}_{1}\\ {\text{of}}_{2}\\ \vdots \\ {\text{of}}_{\text{m}} \end{array}\right]. \end{array}$$

In MFO, moths seek the optimum solution in each iteration, with flames depicting the optimum solution discovered. Location of the flame is then restructured.

**Step 2 (positions of the moths are being updated).**

MFO employs three functions to setup the moths' random placements (*R*), optimal solution (*S*), and stop process (*T*):

(4) $$\begin{array}{c} \text{MFO}=\left(R,S,T\right). \end{array}$$

To setup the moths' location in the optimal position, any random distribution can be utilized. The *R* function's implementation can be written as

(5) $$\begin{array}{c} N\left(A,B\right)=\left(\text{up}\left(A\right)-\text{lo}\left(B\right)\right)*\mathrm{rand}\;\left(\right)+\text{lo}\left(A\right), \end{array}$$

where up and lo are arrays that determine the upper limit and lower limit of the function, respectively. The direction of moths in the optimal position is described using a logarithmic function that is susceptible to the conditions listed as follows:

- The initial point of the spiral should be the moth
- The location of the flame should represent the spiral's ultimate point
- The spiral's reach should not vary more than the problem space

As a result, the *S* represents the movement as shown as follows:

(6) $$\begin{array}{c} S\left(N_{A},{FM}_{B}\right)=D_{A}.e^{ct}.\cos\left(2\pi t\right)+FM_{B}, \end{array}$$

where *c* is a constant used to establish the logarithmic shape, *t* is a random value between 1 and -1, and *D*_*A*_ is the length.

(7) $$\begin{array}{c} D_{A}=\left|{FM}_{B}-N_{A}\right|. \end{array}$$

The spiral path of the moth encircling the flame assures that the optimal solution is explored and utilized. Each cycle sorts the ideal solution (flames) to keep the moths from being stuck in local optima, and it hovers surrounding its associated flame using OF and OM matrix.

**Step 3 (flame update).**

Equation (8) would be used to reduce the number of flames in the MFO algorithm, resulting in the moths solely circling around the optimal solution in the method's final phase.

(8) $$\begin{array}{c} \text{Flame Number}=\text{round}\left(\text{Max}-\text{Cur}*\frac{\text{Max}-\text{Cur}}{\text{Iter}}\right), \end{array}$$

where Cur stands for the existing number of epochs, Max stands for the highest number of flames, and Iter stands for the number of iterations. The solution space developments are balanced by reducing the number of flames.

**Step 4 (termination condition).**

The termination criterion decides when the algorithm should be stopped. The choice of a good termination criterion is critical for the algorithm's correct convergence. The MFO is frequently terminated based on the number of repetitions, the amount of improved performance, and the length of time it has been running.

#### 3.3.2. Feature Extraction by Principal Component Analysis (PCA)

We use the eigenvalue-one criterion to identify the number of meaningful components to keep in the analysis. We were able to keep all components with an eigenvalue larger than 1 as a result of this. As an independent variable, each element accounts for one unit of variation. As a result, components having an eigenvalue larger than one accounted for higher variance compared to individual contributions. Components having eigenvalues less than 1, on the other hand, delivered lesser than the individual and were eliminated.

### 3.4. Classification

The proposed research's subsequent phase is classification. A class label is forecasted for a particular example of input data in classification, which is a predictive modeling (PM) job in ML. PM design is the method of estimating the feature representation from discrete input parameters to discrete independent variables. The primary purpose is to determine which group the additional knowledge corresponds to. There are four classification algorithms incorporated in the proposed research that includes decision tree, SVM, ANN, and KNN.

#### 3.4.1. Decision Tree (DT)

DT is a visual representation of decision taking using an algorithm. A DT is created by asking a yes/no question and then breaking the answer into two parts to lead to another decision. The question is at the node, and the decisions that follow are at the leaves. It may be used to tackle classification and regression problems.

#### 3.4.2. Support Vector Machine (SVM)

SVM is a regulated ML methodology that can tackle classification and regression issues. It may also be utilized to address categorization challenges. Each piece of data is represented as a locus in geometry, without the value of each attribute representing the algorithm's value of a single locus. The categorization is then accomplished by determining the hyperplane that clearly differentiates the 2 groups. An SVM model in high-dimensional space is simply a representation of different groups in a hyperplane. To decrease the error, SVM will create the hyperplane progressively. The goal of SVM is to divide the datasets into groups such that a maximal marginal hyperplane may be identified (MMH). Using these support vectors, we optimize the classifier's margin. If the support vectors are removed, the location of the hyperplane will change.

#### 3.4.3. Artificial Neural Network (ANN)

ANNs are a crude model of how the human brain learns. Neurons, which are in charge of layer generation, make up an ANN. These neurons are also known as tuned factors. The result of each layer is forwarded on to the subsequent layer. Every layer has its own nonlinear activation function, which helps with the process of learning and producing the result. Terminal neurons are another name for the output layer. Each epoch, the weights connected to the neurons and responsible for overall prediction are modified. Various optimizers are incorporated to increase the learning process. Every ANN has objective function that decreases as learning progresses. The best weights for which the cost function gives the best outcomes are then used.

#### 3.4.4. K-Nearest Neighbor (KNN)

KNN is a simplistic, convenient solution for dealing with classification and regression tasks. The KNN technique ensures that the newest scenario and existing scenarios are identical and places the new case in the group that is most close to the original group. KNN is discussed below.

### 3.5. Ensemble Stacking

#### 3.5.1. Stacking

Ensemble learning is a machine learning terminology in which several models are trained to handle the same problem and then integrated to improve results. The main idea is that by correctly combining weak models, we can get more accurate and/or resilient results. A single method may not be able to deliver the best estimate for a given dataset. ML algorithms have limitations, and it is difficult to create a high-accuracy model. The total precision might be enhanced by developing and combining many models. Integrating the results of each system achieves reduced error while keeping generality. This sort of aggregate may be implemented in a variety of ways. Meta-algorithms are a term used in some textbooks to describe such designs.

Stacking is an ML approach used in ensembles. Using a metalearning strategy, it learns how to merge the predictions from two or more ML algorithms. Stacking has the benefit of integrating the characteristics of many high-performing systems to provide predictions that surpass any single model in composition of a classification or regression task.

#### 3.5.2. Logistic Regression

A method for evaluating the probability of a finite result given independent variables is known as logistic regression. A binary outcome is incorporated in the majority common logistic regression methods. To model scenarios with more than 2 distinct outcomes, multinomial logistic regression can be employed. Logistic regression is a powerful statistical method for determining if a fresh data matches well inside a group. Because cyber security components, like threat detection, are categorization issues, logistic regression is a useful analysis technique.

## 4. Results and Discussion

The Cleveland dataset is used to run the proposed architecture. It performs classification using the following steps, namely, preprocessing, feature selection using MFO, feature extraction using PCA, and classification using decision tree, SVM, ANN, and KNN, followed by ensemble staking using logistic regression. The proposed system achieves higher accuracy with reduced computation.

Table 1 shows the description of Cleveland dataset. A heat map helps in visualizing the data present in the dataset.  Figure 2 represents the heat map for Cleveland dataset.  Table 2 represents the instances in the dataset after preprocessing.

For the proposed research, the datasets are divided into two halves: (1) a training part with 70% of the information and (2) a testing part with 30% of the information. Four performance metrics, namely, accuracy, precision, recall, and *F*-measure, are considered in the proposed research. The accuracy rate is obtained through dividing the number of accurate classifications by the total number of classes in the dataset. It is represented in

(9) $$\begin{array}{c} \text{Accuracy}=\frac{\text{Num of correct classes identified}}{\text{Total Num of classes}}. \end{array}$$

Precision, recall, and *F*-measure are estimated using the following equations:

(10) $$\begin{array}{c} \text{Precision}=\frac{\text{True Positive}}{\text{True Positive}+\text{False Positive}}\times 100, \end{array}$$

(11) $$\begin{array}{c} \text{Recall}=\frac{\text{True Positive}}{\text{True Positive}+\text{False Negative}}\times 100, \end{array}$$

(12) $$\begin{array}{c} \text{F}‐\text{Measure}=2\times \frac{\text{Precision}\times \text{Recall}}{\text{Precision}+\text{Recall}}\times 100. \end{array}$$

Accuracy, precision, recall, and *F*-measure should improve over period.  Table 3 shows the research findings without preprocessing and with preprocessing technique like noise removal by removing missing values, normalization using min-max, normalization using *Z*-score, and combined results. Various metaheuristic algorithms are applied for various applications [34–39].  Table 4 displays the results of experimentation using several feature selection strategies such as the genetic algorithm, particle swarm optimization, and Moth-Flame Optimization. The proposed method using MFO achieves the best result when compared with other techniques.  Table 5 displays the results of the experiment of several feature extraction strategies, with the PCA employed in the proposed method producing the best results in comparison with other approaches.  Figure 3 depicts a comparison of preprocessing methods.

Table 6 shows the experimental classification approaches like DT, SVM, ANN, and KNN. The result after applying ensemble stacking using logistic regression produces the best results than applying individual models. When compared to previous strategies, the current technique employing MFO delivers superior results.

Table 7 shows the result of comparison of the proposed method with various existing techniques.  Figure 4 shows the comparison with various feature selection and feature extraction techniques.  Figure 5 shows the comparison with several state-of-art methodologies. The recommended strategies produce superior performance in the aspects of accuracy, precision, recall, and *F*-measure.

## 5. Conclusions and Future Work

Many lives are saved to healthcare monitoring and prediction technologies, especially when patients are placed distant. The classifier's objective was to determine whether a patient had cardiovascular disease or not. When system resources must be considered, using all functionalities is not possible. In this work, we utilized dimensionality reduction methods to enhance the original collected data. Classification was performed using decision trees, SVM, ANN, and KNN, and ensemble stacking called logistic regression helped in achieving the best results from the various classification models. Our technology may be used to evaluate large volumes of data and discover the risk variables associated with various diseases in a variety of real-world applications or in other medical diagnoses. We intend to test our strategy on a larger dataset and analyze a different disease using alternative feature selection strategies. Our key limitation is that the limited sample size makes it difficult to generalize these findings to heart disease. In further work, we intend to expand the dataset to which our method will be used and analyze more diseases using various feature selection methods.

## Figures and Tables

**Figure 1:** Schematic diagram of proposed system.

**Figure 2:** Heat map of Cleveland dataset.

**Figure 3:** Comparison of preprocessing techniques.

**Figure 4:** Comparison of (a) feature selection techniques and (b) feature extraction technique.

**Figure 5:** Comparison of various state-of-art methods.

**Algorithm 1:** Algorithm of KNN.

**Table 1:** Cleveland dataset used for the proposed system.

Name	Cleveland
Total # of instances	303
Number of attributes	75
Omitted values	Yes
Dataset type	Multivariate
Attribute type	Categorical, integer, real
Tasks performed	Classification

**Table 2:** Instances in the dataset after preprocessing.

Name	Instances present	With HD	Without HD
Cleveland	283	157 (55%)	126 (45%)

**Table 3:** Experimental results of preprocessing technique.

S. no	Method	Precision (%)	Recall (%)	*F*-measure (%)	Accuracy (%)
1	No preprocessing	80	80	81	79
2	Noise removal	82	80	86	85
3	Normalization using min-max	86	84	80	87
4	Normalization using *Z*-score	87	85	86	86
5	Combining 2, 3, and 4	90	89	89	91

**Table 4:** Experimental results of feature selection approach.

S. no	Methodology	Precision (%)	Recall (%)	*F*-measure (%)	Accuracy (%)
1	Genetic algorithm	82	81	76	81
2	Particle swarm optimization	87	86	84	89
3	Moth-Flame Optimization	90	87	87	91

**Table 5:** Experimental results of feature extraction approach.

S. no	Methodology	Precision (%)	Recall (%)	*F*-measure (%)	Accuracy (%)
1	Linear discriminant analysis (LDA)	81	79	73	80
2	Nonnegative matrix factorization (NMF)	80	83	84	85
3	Principal component analysis (PCA)	90	86	87	90

**Table 6:** Experimental results of classification approach.

S. no	Methodology	Precision (%)	Recall (%)	*F*-measure (%)	Accuracy (%)
1	DT	94	95	98	98
2	SVM	96	98	98	99
3	ANN	98	94	97	98
4	KNN	97	97	98	96
5	Ensemble stacking	98	98	99	99

**Table 7:** Evaluation with other existing studies.

S. no	Approaches	Precision (%)	Recall (%)	*F*-measure (%)	Accuracy (%)
1	Miao et al. [40]	81	71	80	80
2	Naidu and Rajendra [41]	80	85	82	85
3	Shamosollahi et al. [42]	92	90	90	92
4	Hungarian dataset	93	91	95	94
5	Proposed method (Cleveland dataset)	98	98	99	99

## Data Availability

The authors confirm that the data supporting the proposed work are taken from publically available datasets.
